RETRACTED

# Expression of Serum Omentin, CTRP9, and Vaspin in Patients with Polycystic Ovary Syndrome

**DOI:** 10.1155/2022/1862404

**Published:** 2022-08-17

**Authors:** Yuhong Wang, Ning Liu, Jing Lu, Liping Yang, Changyan Wang, Jing Chen, Wenliang Chang

**Affiliations:** Department of Reproductive Medicine, Handan Central Hospital, Handan 056000, Hebei, China

## Abstract

**Objective:**

To explore the relationship between serum omentin, C1q/tumor necrosis factor-related protein-9 (CTRP9), and visceral fat-specific serine protease inhibitor (vaspin) levels in different phenotypes in patients with polycystic ovary syndrome (PCOS).

**Methods:**

One hundred PCOS patients treated at our hospital's clinic of reproductive medicine were chosen and included into the research group, and 100 healthy women who came for physical examination during the same time period were included into the control group. According to the definition of obesity by the WHO (body mass index (BMI) ≥25 kg/m^2^), 100 patients with PCOS were equally divided into obese (study group A) and nonobese (study group B) groups. 100 healthy women were also divided into obese (control group A) and nonobese (control group B) groups with 50 patients each. Comparison among the 4 groups was performed in factors/indicators including the serum omentin, CTRP9, and vaspin levels and biochemical indexes (triglyceride (TG), total cholesterol (TC), high density lipoprotein cholesterol (HDL-C), low density lipoprotein cholesterol (LDL-C), fasting insulin (FINS), total testosterone, and homeostasis model assessment of insulin resistance (HOMA-IR) levels), and the correlation analysis was conducted with omentin, CTRP9, and vaspin.

**Results:**

There was no significant difference in age, TG, TC, and LDL-C among the 4 groups (*P* > 0.05). The BMI, WHR, HDL-C, and omentin of the obese phenotype were significantly different from those of the nonobese phenotype (*P* < 0.05). Among the four groups, FINS, HOMA-IR, and vaspin in group A (obesity) was the highest, and the control group B (nonobese) was the lowest. There was no significant difference in the levels of study group B (nonobese) and control group A (obesity). The level of CTRP9 in the study group was significantly lower than that in the control group (*P* < 0.05). Taking serum omentin, CTRP9, and vaspin levels of patients in the study group as dependent variables, Pearson correlation analysis showed that the omentin level was negatively correlated with BMI, WHR, FINS, TG, TC, LDL-C, HOMA-IR, and TT levels (*P* < 0.05) and was positively correlated with the HDL-C level (*P* < 0.05); CTRP9 level was negatively correlated with BMI, TC, and HOMA-IR (*P* < 0.05) and was not correlated with age, WHR, FINS, TG, HDL-C, LDL-C, HOMA-IR, and TT levels. The vaspin level was positively correlated with BMI, WHR, FINS, TG, TC, LDL-C, HOMA-IR, and TT levels (*P* < 0.05) and negatively correlated with HDL-C levels (*P* < 0.05) and was not correlated with age.

RETRACTED

**Conclusion:**

When compared with healthy people, PCOS patients have higher serum vaspin levels and lower CTRP9 levels; BMI, TC, LDL-C, FINS, TG, total testosterone, HDL-C levels, waist-to-hip ratio, and HOMA-IR are all closely related to serum vaspin and CTRP9 levels; increasing serum CTRP9 levels and decreasing vaspin levels help to slow progress and promote prognosis of the disease. Serum omentin level is connected with the obesity index but not with PCOS.

## 1. Introduction

Polycystic ovary syndrome (PCOS) is one of the most common reproductive and endocrine disorders in gynecology. With complex pathogenesis, it is characterized by chronic anovulation and hyperandrogenism [1, 2]. Typical symptoms such as menstrual disorder, infertility, obesity, and others could have serious impact on the physical and psychological health of women at reproductive age. And, with the progress of the disease, it would possibly raise the risk of endometrial cancer, gestational diabetes, and hyperlipidemia. About 5%–10% of reproductive women are affected by PCOS, 15% to 20% of the infertile women was diagnosed with PCOS. In addition to the disorder of sex hormone metabolism, most patients with PCOS also disorder of glucose and lipid metabolism [3–5].

In modern western medicine, PCOS is commonly treated with diane-35, an oral contraceptive medicine. Hyperandrogenism symptoms can be effectively attenuated but is prone to recurrence after withdrawal. For infertile women of reproductive age with PCOS, clomiphene citrate (CC) or human chorionic gonadotropin (HCG) is prescribed orally to promote ovulation, with the advantages of low cost and fewer by-effects. But research showed that the probability of pregnancy for patients treated with CC or HCG is only about a half. As for surgery, it comes with short term effects and high risk of recurrence, with certain damage to the body and high incidence of postoperative adhesion [6, 7]. In recent years, more and more researchers looked into the effect of traditional Chinese medicine (TCM) on PCOS. It was found to be with fewer by-effects, higher security, and longer efficacy. TCM scholars found that PCOS is similar to diseases in TCM gynecology like “menstrual blood melting down or dripping,” “menstruation delay,” and “amenorrhea.” Most TCM doctors believe that the occurrence of the disease is inseparable from the liver, spleen, and kidney. Weak kidney impedes development of human body, spleen deficiency causes phlegm and dampness, and liver-Qi stagnation leads to blood stasis; then, the normal operation of blood and *Qi* would be disrupted and so came the disease [8, 9]. As the TCM wisdom holds “superior doctors cure diseases before external symptom shows,” early stage prevention and diagnosis is of utterly importance.

RETRACTED

In clinical settings, exclusionary diagnosis is commonly used to clarify patients' condition based on clinical symptoms and ultrasonography image. However, the condition of PCOS patients is fairly complex for highly varied clinical symptoms and ultrasound imaging presentations, making it readily mistaken with other conditions, resulting in missed diagnosis and misdiagnosis [10, 11]. Therefore, it is of great clinical significance to seek PCOS serum markers with high sensitivity and specificity. Multiple alternatives have been reported to predict PCOS, such as anti-Müllerian hormone (AMH) level, higher blood urea nitrogen to albumin ratio (BAR) (>7.83) for long-term mortality in AMI patients, elevated ADMA, CRP, Hcy, PAI-1, VEGF, ANGPTL6, and endotrophin level [12–14].

Current studies have concluded that serum omentin is involved in regulating and maintaining the balance of glucose and lipid metabolism from changes in the levels of serum lactones, adiponectin, omentin, and other indicators in patients with PCOS [15]. Other research believes omentin, as a hormone released by the omental tissue that regulates metabolism and immunological response, may be implicated in the development of insulin resistance and hence the pathological process of PCO [16]. C1q/tumor necrosis factor-related protein 9 (CTRP9) is an adipokines that synthesize and secrete adipose tissue, which can protect the myocardium and blood vessels, regulate metabolism, and exert an anti-inflammatory function [17, 18]. Vaspin is a serine protease inhibitor first identified by Hida et al. in 2005. It is involved in the process of glucose and lipid metabolism in the body and is closely related to endocrine function [19, 20]. Vaspin gene polymorphisms have been discovered to be strongly related with diabetes and cardiovascular disease in studies. Currently, few research focused on the expression of serum omentin, CTRP9, and vaspin in PCOS patients. This study will investigate the relationship between serum omentin, CTRP9, vaspin, glucose, and lipid metabolism, *T*, body mass index (BMI), and islet function in patients with PCOS.

## 2. Research Objects and Methods

### 2.1. Research Objects

From April 2019 to April 2021, 100 PCOS patients treated at our hospital's clinic of reproductive medicine were chosen and included into the research group, and 100 healthy women who came for physical examination during the same time period were included into the control group. According to the definition of obesity by the WHO (body mass index (BMI) ≥25 kg/m^2^), 100 patients with PCOS were equally divided into obese (study group A) and nonobese (study group B) groups. The 100 healthy women were also divided into obese (control group A) and nonobese (control group B) groups with 50 patients each. The age of the control group was 22–54 years, with an average of 35.42 ± 7.51 years. The age of the study group ranged from 21 to 52 years, with an average of 34.94 ± 8.07 years.

RETRACTED

Inclusion criteria for the study group: (1) met the diagnostic criteria in the “Chinese Diagnostic Guidelines for Polycystic Ovary Syndrome” [21]; (2) had no history of diabetes, cardiovascular disease, and hypertension; (3) had not taken insulin sensitizers and steroid hormone drugs in the past 3 months; (4) signed the informed consent.

Inclusion criteria for the control group: (1) with normal menstrual cycle; (2) without polycystic ovarian changes (confirm through ultrasound examination); (3) with normal basal sex hormone levels.

The exclusion criteria for both the study group and the control group were as follows: (1) without a complete uterus and ovary; (2) in acute phase of systemic diseases; (3) with other endocrine diseases, tumors, and cardiovascular diseases. All those research objects have been informed and been required to sign the informed consent before inclusion. Patients in study group and healthy women in control group were fully informed of the purpose of the study, and the experiment was authorized by the ethics committee of Handan Central Hospital (registration number: HD-7768-19). All procedures comply with the ethical guidelines of the Declaration of Helsinki on clinical research.

### 2.2. Experimental Method

#### 2.2.1. Basic Data Collection

Basic information of all subjects, including age, BMI, waist-to-hip ratio (WHR) (BMI = weight/height (kg/m2); WHR = waist/hip (cm/cm)); systolic blood pressure (SBP) and diastolic blood pressure (DBP), was measured 3 times to obtain the average value.

### 2.3. Biochemical Indexes Measurement

On the morning of the fourth day of a menstrual cycle (any time for amenorrhea patients), 5 ml of fasting venous blood was drawn from all subjects to determine serum omentin, CTRP9, and vaspin levels and biochemical indicators (triglyceride (TG), total cholesterol (TC), high density lipoprotein cholesterol (HDL-C), low density lipoprotein cholesterol (LDL-C), fasting insulin (FINS), total testosterone, and homeostasis model assessment of insulin resistance (HOMA-IR)). Among them, the levels of serum omentin, CTRP9, and vaspin were determined using an enzyme-linked immunosorbent assay, blood lipids were determined by a fully automated biochemical detector, total testosterone, and FINS levels were determined using electrochemiluminescence, and plasma glucose level was measured through the glycokinase method. HOMA-IR = fasting blood glucose (FBG)* × *FINS/22.5.

RETRACTED

### 2.4. Outcome Indicators

The levels of omentin, CTRP9, and vaspin in serum were compared amongst the four groups.

### 2.5. Statistical Analysis

All data were processed by SPSS 22.0, measurement data were expressed as *x* ± *s*, and independent samples *T* test was used for comparison between groups, while one-way ANOVA was used for comparison amongst multiple groups. Relationship between indicators was determined by Pearson linear correlation and multiple linear regression analysis. *P* < 0.05 was assumed as statistically significant.

## 3. Results

### 3.1. Comparison of Clinical Data and Metabolism-Related Indicators among the Four Groups

There was no significant difference in age, TG, TC, and LDL-C among the 4 groups (*P* > 0.05). The obese phenotype's BMI, WHR, HDL-C, and omentin levels were considerably higher than those of the nonobese phenotype (*P* < 0.05). FINS, HOMA-IR, and vaspin levels were the highest in group A (obese), and the lowest in control group B (nonobese), with no significant difference between study group B (nonobese) and control group A (obese). CTRP9 level of the study group was considerably lower than of the control group (*P* < 0.05), as shown in Table 1.

### 3.2. Analysis of Factors Related to Serum Omentin, CTRP9, and Vaspin Levels

With serum omentin, CTRP9, and vaspin levels as dependent variables, Pearson correlation analysis revealed that the omentin level was negatively correlated with BMI, WHR, FINS, TG, TC, LDL-C, HOMA-IR, and TT levels but positively correlated with the HDL-C level (*P* < 0.05); the CTRP9 level was negatively correlated with BMI, TC, and HOMA-IR (*P* < 0.05) and was not correlated with age, WHR, FINS, TG, HDL-C, LDL- C, HOMA-IR, and TT levels. The vaspin level was positively correlated with BMI, WHR, FINS, TG, TC, LDL-C, HOMA-IR, and TT levels (*P* < 0.05) and negatively correlated with HDL-C levels (*P* < 0.05) and was not correlated with age (see Table 2).

## 4. Discussion

PCOS, one of the most common reproductive endocrine diseases in women, is often manifested as ovulatory dysfunction, hyperandrogen status, hyperinsulinemia, and ovarian polycystic changes [22]. Though its pathology has yet to be fully understood, most scholars believe that lipid metabolism, heredity, body hormone level, and other factors are engaged [23, 24]. Data shows that 30%∼60% of PCOS patients are obese, 50%∼70% of PCOS patients are also diagnosed with insulin resistance, and insulin resistance may be the central link or initial factor of the disease. The development of insulin resistance is related to the conduction defect of insulin signal pathway [25, 26]. It is reported that, in recent years, the population diagnosed with PCOS becomes increasingly larger and younger, posing great hazard on the physical and mental health of women of childbearing age. However, due to the complexity and diversity of PCOS, its pathogenic causes and mechanisms are still not clear, and some studies believe that it is related to genetic, endocrine, metabolic, immune, environmental, mental and psychological factors. PCOS is a refractory disease and cannot be completely cured for now. In clinical practice, symptomatic treatments such as ovulation promotion, androgen reduction, and insulin resistance alleviation are mainly used, and surgical treatment is adopted when necessary [27, 28].

RETRACTED

Western medicine has not clarified the exact pathogenesis of PCOS, but genetic and environmental factors are considered to be the possible directions for exploration. According to the clinical symptoms of patients with PCOS, western medicine applies symptomatic treatment. For example, estrogen and progesterone are used to regulate women's menstrual cycle, androgen lowering therapy is adopted for patients with high androgen, and ovulation promotion and ovarian drilling are applied to patients with fertility requirements [29, 30]. In traditional Chinese medicine, there is no related record of “polycystic ovary syndrome,” but its clinical manifestations such as irregular menstruation, rare hair, late closure, amenorrhea, and irregular uterine bleeding relate it to diseases like “menstruation delay,” “amenorrhea,” and “infertility.” Clinical manifestations of this disease are diverse, and the dialectical classification is complex. So far, a unified dialectical treatment standard has not been reached. Most doctors think that the disease is mainly related to the dysfunction of an axis from kidney–Tiankui (menstruation)—Chong and Ren Meridians–and finally to uterine. Kidney deficiency harms menstruation, spleen deficiency induces endogenous wet and turbidities, and liver stagnation impedes free flow of Qi and blood. As time goes by, wet, phlegm, blood stasis, and other pathological products accumulates in the body and will eventually block Chong and Ren meridians and uterine if not cured in time and then lead to PCOS. Doctors hold different dialectical views on treatment, but the methods they adopted are invariably from the basic pathogenesis of viscera deficiency and the intermingled deficiency and excess [31, 32].

RETRACTED

More and more studies have shown that PCOS is not only a reproductive system dysfunction but rather a complex multisystem syndrome [33, 34]. Despite advances in PCOS related research, the cause of the condition remains unknown. People tend to focus on menstruation and fertility, thus overlooking metabolic problems and insulin resistance (IR) in patients. IR and the dysfunction of hypothalamic-pituitary-gonadal axis could be two core links in the progress of PCOS. Patients with PCOS are faced with higher risks of metabolic abnormalities, dyslipidemia, and cardiovascular problems, but opinions still varied on whether adipokines are related to the occurrence and development of gynecological endocrine diseases.

Adipose tissue is an endocrine organ that can perform autocrine and paracrine, store energy, and form an intricate metabolic-neuroendocrine-immune network. Serum vaspin and CTRP9 are adipokines most commonly seen in clinical studies on obesity and cardiovascular diseases [35]. As studies go deeper, it is found out that adipose tissue can not only store energy but also produce hormones (called adipokines). In other words, adipose tissue performs endocrine function. Vaspin, a member of the serine protease inhibitor family, is found in visceral adipose tissue and exhibits insulin-sensitizing property. Elevated serum vaspin concentration is associated with obesity and altered insulin sensitivity in humans. As reported in previous studies, the serum vaspin level, if abnormally elevated, can induce abnormal lipid metabolism, and elevated levels of hormones in patients can lead to hormone regulation disorder and thus increase its content [36]. In animal experiments, Bongrani et al. [37] found that when the body weight and insulin resistance index of obese diabetic rats rose, their serum vaspin levels also increased, and vice versa. After insulin sensitizer treatment, their serum vaspin levels markedly increased. Thus, serum vaspin may have a role in insulin sensitivity. The serum vaspin level in PCOS patients was higher than that in healthy subjects, indicating its role of a indicator for clinical diagnosis of PCOS, and the increase in its level may be the body's compensatory response to the glucose metabolism disorder and insulin resistance. In addition, this study also found the following correlations between serum vaspin and lipid metabolism and obesity of PCOS patients: serum vaspin is positively correlated with BMI, WHR, FINS, TG, TC, LDL-C, HOMA-IR, and TT levels and negatively correlated with HDL-C (*P* < 0.05). A possible reason may be that the increase of body fat content stimulates adipose tissue to a certain extent, prompting it to secrete vaspin, which contributes to fat deposit in a compensatory manner or it may be related to the compensatory increase of vaspin expression in obesity.

RETRACTED

Adiponectin is a cytokine negatively correlated with obesity. Secreted and synthesized by adipocytes, it has many biological effects such as antiatherosclerosis, antidiabetes, anti-inflammatory, and antiapoptosis [38]. The CTRPs family, discovered clinically in recent years, is highly homological to adiponectin. Among them, CTRP9 and can be used as an indicator to reflect the body's insulin sensitivity [39]. This study showed that the CTRP9 level was negatively correlated with BMI, TC, and HOMA-IR, but had no correlation with age, WHR, FINS, TG, HDL-C, LDL-C, HOMA-IR, and TT levels. As for the reason behind, we think that CTRP9 level may affect liver cholesterol synthesis and decomposition or blood sugar tolerance, resulting in local oxidative stress injury or local stress injury caused by blood lipid metabolism disorder, thereby promoting local ovarian epithelial endocrine functional disorders in PCOS patients, inhibiting ovulation and inducing excessive androgen secretion and further facilitating progress of PCOS in patients.

Since the lowering of the omentin level is related to insulin resistance and obesity, we speculated that omentin plays a role in the occurrence and development of PCOS [40]. In this study, serum omentin in PCOS patients was found to be significantly lower than that in normal people of the control group, and that omentin level was negatively correlated with BMI, WHR, FINS, TG, TC, LDL-C, HOMA-IR, and TT levels and positively correlated with the HDL-C level. Thus, the speculation was supported.

Due to objective factors like funds, time and complexity, and diversity of the disease, this study included relatively a small number of patients with limited observation indicators, short time of observation, and follow-up visits, from which the evaluation of clinical effects was not comprehensive. The absence of animal tests means the action mechanism of relevant drugs could not be further explored.

Multicenter clinical research with expanded sample size, double-blind comparison, longer time of treatment, observation, and follow-up visits, standardize and accurate observation indicators, and animal tests when necessary to explore the pharmacological mechanism is supposed to be the future direction.

In conclusion, PCOS patients present higher serum vaspin levels and lower CTRP9 levels when compared with healthy people; BMI, TC, LDL-C, FINS, TG, total testosterone, HDL-C levels, waist-to-hip ratio, and HOMA- IR are closely related to serum vaspin and CTRP9 levels; increasing serum CTRP9 level and reducing vaspin level can help slow the progress of PCOS and promote disease prognosis. Serum omentin level is associated with the obesity index but not with PCOS.

RETRACTED

## Figures and Tables

**Table 1:** Comparison of clinical data and metabolism-related indexes of the four groups ($\bar{x}$ ±*s*).

Groups	*n*	Age (year)	BMI (kg/m^2^)	WHR	FINS (mIU/L)	
Study group A (obesity)	50	34.63 ± 6.09	27.84 ± 3.87^a^	0.97 ± 0.07^a^	24.93 ± 16.37^ac^	
Study group B (nonobesity)	50	33.81 ± 7.11	20.69 ± 1.62	0.84 ± 0.08	10.63 ± 6.92^d^	
Control group A (obesity)	50	35.25 ± 7.48	27.33 ± 4.25^b^	0.96 ± 0.06^b^	10.60 ± 6.84^b^	
Control group B (nonobesity)	50	34.66 ± 7.50	19.81 ± 1.60	0.82 ± 0.05	4.22 ± 1.91	
*F*		1.326	63.269	13.731	35.536	
*P*		0.294	≤0.001	≤0.001	≤0.001	

Groups	n	TG (mmol/L)	TC (mmol/L)	HDL-c (mmol/L)	LDL-c (mmol/L)	

Study group A (obesity)	50	2.84 ± 0.89	4.67 ± 1.13	1.11 ± 0.24^a^	3.32 ± 0.61	
Study group B (nonobesity)	50	1.57 ± 1.08	4.62 ± 1.24	1.19 ± 0.35	2.79 ± 0.55	
Control group A (obesity)	50	2.23 ± 1.46	4.57 ± 0.96	1.13 ± 0.21^b^	3.22 ± 0.78	
Control group B (nonobesity)	50	1.58 ± 0.92	4.38 ± 0.73	1.24 ± 0.35	2.97 ± 0.92	
*F*		2.132	0.656	3.679	1.673	
*P*		0.110	0.592	0.015	0.179	

Groups	n	HOMA-IR	TT (mmol/L)	Omentin (pg/L)	CTRP9 (ng/L)	Vaspin (μg/L)

Study group A (obesity)	50	6.37 ± 1.52^ac^	1.47 ± 0.62^c^	42.87 ± 19.52^a^	239.31 ± 36.17^c^	0.63 ± 0.44^ac^
Study group B (nonobesity)	50	2.31 ± 1.57^d^	1.41 ± 0.53^d^	111.23 ± 34.74	241.76 ± 42.73^d^	0.45 ± 0.34^d^
Control group A (obesity)	50	2.26 ± 1.55^b^	1.04 ± 0.87^b^	45.91 ± 18.54^b^	463.58 ± 64.72	0.33 ± 0.31^b^
Control group B (nonobesity)	50	0.91 ± 0.38	0.93 ± 0.47	115.28 ± 33.78	461.39 ± 55.45	0.13 ± 0.10
*F*		22.341	4.131	60.308	206.516	6.782
*P*		≤0.001	≤0.001	≤0.001	≤0.001	≤0.001

**Table 2:** Analysis of related influencing factors of serum omentin, CTRP9, and vaspin levels ($\bar{x}$ ± *s*).

Indexes	Omentin		CTRP9		Vaspin	
	*r*	*P*	*r*	*P*	*r*	*P*
Age	−0.356	0.021	0156	0.231	0.023	0.136
BMI	−0.913	0.007	−0.323	0.008	0.211	0.021
WHR	−0.640	0.041	0.055	0.673	0.197	0.003
FINS	−0.529	0.033	−0.079	0.553	0.204	0.017
TG	−0.641	0.006	0.040	0.905	0.192	0.007
TC	−0.722	0.009	−0.341	0.010	0.191	0.023
HDL-C	0.917	0.034	−0.085	0.512	−0.212	0.031
LDL-C	−0.338	0.027	−0.071	0.575	0.231	0.019
HOMA-IR	−0.402	0.005	−0.309	0.021	0.217	0.023
TT	−0.715	0.039	−0.112	0.059	0.209	0.025

## Data Availability

All data generated or analysed during this study are included in this published article.

## References

[1] Ajmal N., Khan S. Z., Shaikh R. (2019). Polycystic ovary syndrome (PCOS) and genetic predisposition: a review article. *European Journal of Obstetrics & Gynecology and Reproductive Biology X*.

RETRACTED

[2] Kamenov Z., Gateva A. (2020). Inositols in PCOS. *Molecules*.

[3] Khan M. J., Ullah A., Basit S. (2019). Genetic basis of polycystic ovary syndrome (PCOS): current perspectives. *The Application of Clinical Genetics*.

[4] Delcour C., Robin G., Young J., Dewailly D. (2019). PCOS and Hyperprolactinemia: what do we know in 2019?. *Clinical Medicine Insights: Reproductive Health*.

[5] Patel S. (2018). Polycystic ovary syndrome (PCOS), an inflammatory, systemic, lifestyle endocrinopathy. *The Journal of Steroid Biochemistry and Molecular Biology*.

[6] Wang Y., Xing Y., Xing Y. U. (2022). Clinical observation on the treatment of obese polycystic ovary syndrome with Bushen Huatan Decoction combined with acupunctur. *China Family Planning and Obstetrics*.

[7] Lipei J. (2022). Clinical study of Bushen Huayu Recipe combined with western medicine in the treatment of polycystic ovary syndrome infertility. *New Chinese Medicine*.

[8] Song W., Yan J. (2022). Clinical effect of Bushen Huayu Recipe combined with moxibustion in the treatment of ovulatory infertility with blood stasis type polycystic ovary syndrome. *Journal of Clinical Rational Medicine*.

[9] Xie C., Zhao Y., Zhang A. (2022). Ultrasound observation of uterine artery blood flow in patients with polycystic ovary syndrome treated with Jianpi Huatan Formula. *Journal of Hubei University of Traditional Chinese Medicine*.

[10] Witchel S. F., Teede H. J., Peña A. S. (2020). Curtailing PCOS. *Pediatric Research*.

[11] Otto-Buczkowska E., Grzyb K., Jainta N. (2018). Polycystic ovary syndrome (PCOS) and the accompanying disorders of glucose homeostasis among girls at the time of puberty. *Pediatric Endocrinology, Diabetes and Metabolism*.

[12] Guney G., Taskin M. I., Baykan O. (2021). Endotrophin as a novel marker in PCOS and its relation with other adipokines and metabolic parameters: a pilot study. *Therapeutic Advance Endocrinology Metabolism*.

[13] Elci E., Kaya C., Cim N., Yildizhan R., Elci G. G. (2017). Evaluation of cardiac risk marker levels in obese and non-obese patients with polycystic ovaries. *Gynecological Endocrinology*.

[14] Cengiz H., Ekin M., Dagdeviren H., Yildiz Ş, Kaya C., Kanawati A. (2014). Comparison of serum anti-Müllerian hormone levels in normal weight and overweight-obese adolescent patients with polycystic ovary syndrome. *European Journal of Obstetrics & Gynecology and Reproductive Biology*.

[15] Watanabe T., Watanabe-Kominato K., Takahashi Y., Kojima M., Watanabe R. (2017). Adipose tissue-derived omentin-1 function and regulation. *Comprehensive Physiology*.

RETRACTED

[16] Lin S., Li X., Zhang J., Zhang Y. (2021). Omentin-1: protective impact on ischemic stroke via ameliorating atherosclerosis. *Clinica Chimica Acta*.

[17] Rezabakhsh A., Sadeghpour Y., Ghaderi S., Rahbarghazi R., Geranmayeh M. H. (2020). CTRP9: an emerging potential anti-aging molecule in brain. *Cellular Signalling*.

[18] Lei S., Chen J., Song C. (2021). CTRP9 alleviates foam cells apoptosis by enhancing cholesterol efflux. *Molecular and Cellular Endocrinology*.

[19] Kurowska P., Mlyczyńska E., Dawid M. (2021). Review: vaspin (SERPINA12) expression and function in endocrine cells. *Cells*.

[20] Kurowska P., Mlyczyńska E., Dawid M., Grzesiak M., Dupont J., Rak A. (2020). The role of vaspin in porcine corpus luteum. *Journal of Endocrinology*.

[21] Lou D., Guo H. (2022). Therapeutic effect of Bushen Huoxue Recipe on polycystic ovary syndrome-induced ovulatory infertility patients with kidney deficiency and blood stasis syndrome. *World Journal of Integrative Medicine*.

[22] Rodriguez Paris V., Bertoldo M. J. (2019). The mechanism of androgen actions in PCOS etiology. *Medical Science*.

[23] Wang Y. (2022). Analysis of the curative effect of self-made Bushen Shugan Qingfei Decoction in the treatment of polycystic ovary syndrome. *Chinese Journal of Clinical Research*.

[24] Gong S., Sun X., Wang J. (2022). Observation on the clinical efficacy of Gubentongjing prescription in the treatment of obese polycystic ovary syndrome. *Clinical Research in Traditional Chinese Medicine*.

[25] Yin S., Wang K., Pang X. (2022). Clinical effect of traditional Chinese medicine prescription in the treatment of obesity with polycystic ovary syndrome. *China Medical Science*.

[26] Yang Y., Wan L., Ding C. (2022). Effects of Bushen Huoxue Recipe on follicular development and pregnancy in patients with polycystic ovary syndrome. *New Chinese Medicine*.

[27] Lv X., Liu J., Yang H. (2022). Observation on the effect of self-made Bushen and Progest Recipe combined with letrozole in the treatment of infertility with polycystic ovary syndrome due to kidney-yin deficiency. *Shandong Medicine*.

[28] Xu J., Cao L., Chen Y. (2022). Observation on the effect of soothing liver and spleen therapy on autoimmune thyroid disease complicated with obesity polycystic ovary syndrome. *Modern Diagnosis and Treatment*.

[29] Ye Y., Huang S. (2022). Clinical observation of Cai’s polycystic formula combined with letrozole in the treatment of infertility with polycystic ovary syndrome due to kidney deficiency and phlegm stasis. *Zhejiang Journal of Traditional Chinese Medicine*.

[30] Li R. (2022). Clinical efficacy of self-made Bushen Jianpi recipe combined with Nuangongyunzi capsules in the treatment of polycystic ovary syndrome. *Practical Chinese and Western Medicine*.

RETRACTED

[31] Wang X. (2022). Effect of Bushen Huoxue Qutan Recipe combined with desogestrel and ethinyl estradiol tablets in the treatment of polycystic ovary syndrome and its effect on endometrial thickness. *China Medical Innovation*.

[32] Dong Y., Cheng X., Zhou J. (2021). Observation on the efficacy of Bushen Jianpi recipe combined with letrozole in the treatment of infertility with polycystic ovary syndrome. *Hainan Medical Journal*.

[33] Wang L., Zhou J., Gober H. J. (2021). Alterations in the intestinal microbiome associated with PCOS affect the clinical phenotype. *Biomedicine & Pharmacotherapy*.

[34] Chen B., Xu P., Wang J., Zhang C. (2019). The role of MiRNA in polycystic ovary syndrome (PCOS). *Gene*.

[35] Wang J., Chen Z., Guan Z. (2021). Vaspin deficiency failed to promote the proliferation of BMSCs in osteoarthritis. *International Journal of Rheumatic Diseases*.

[36] Akyol A., Demirkıran D., Akdag S. (2021). Serum vaspin levels and carotid intima-media thickness in predialysis patients. *European Journal of Clinical Investigation*.

[37] Bongrani A., Mellouk N., Ramé C. (2021). Vaspin, a novel adipokine in woman granulosa cells physiology and PCOS pathogenesis?. *Journal of Endocrinology*.

[38] Song C. X., Chen J. Y., Li N., Guo Y. (2021). CTRP9 enhances efferocytosis in macrophages via MAPK/Drp1-Mediated mitochondrial fission and AdipoR1-induced immunometabolism. *Journal of Inflammation Research*.

[39] Yang M. M., Balmert L. C., Marangoni R. G. (2021). Circulating CTRP9 is associated with severity of systemic sclerosis-associated interstitial lung disease. *Arthritis Care & Research*.

[40] Gatev T., Byalkova V., Poromanski I., Velikova T., Vassilev D., Kamenov Z. (2022). Omentin-1 and diabetic foot. *The International Journal of Lower Extremity Wounds*.

